This article has been retracted.

# Applications of Neural Network-Based Plan-Cancer Method for Primary Diagnosis of Mesothelioma Cancer

**DOI:** 10.1155/2023/3164166

**Published:** 2023-02-04

**Authors:** Dhiraj Kapila, Sarika Panwar, M. K. Mohan Maruga Raja, Tamal Mondal, Shaik Mohammad Rafi, Suryabhan Pratap Singh, Bhupendra Kumar

**Affiliations:** ^1^Department of Computer Science & Engineering, Lovely Professional University, Phagwara, Punjab, India; ^2^Department of Electronics and Telecommunication Engineering, AISSMS's Institute of Information Technology, Pune, India; ^3^Parul Institute of Pharmacy & Research, Parul University, Vadodara, Gujarat, India; ^4^Department of Botany, Hiralal Mazumdar Memorial College for Women, Dakshineswar, Kolkata 700035, India; ^5^Department of Computer Science and Engineering, Sri Mittapalli College of Engineering, Guntur, Andhra Pradesh, India; ^6^Information Technology, Institute of Engineering and Technology, Deen Dayal Upadhyaya Gorakhpur University, Gorakhpur, India; ^7^Debre Tabor University, Debre Tabor, Ethiopia

## Abstract

“Malignant mesothelioma (MM)” is an uncommon although fatal form of cancer. The proper MM diagnosis is crucial for efficient therapy and has significant medicolegal implications. Asbestos is a carcinogenic material that poses a health risk to humans. One of the most severe types of cancer induced by asbestos is “malignant mesothelioma.” Prolonged shortness of breath and continuous pain are the most typical symptoms of the condition. The importance of early treatment and diagnosis cannot be overstated. The combination “epithelial/mesenchymal appearance of MM,” however, makes a definite diagnosis difficult. This study is aimed at developing a deep learning system for medical diagnosis MM automatically. Otherwise, the sickness might cause patients to succumb to death in a short amount of time. Various forms of artificial intelligence algorithms for successful “Malignant Mesothelioma illness” identification are explored in this research. In relation to the concept of traditional machine learning, the techniques support “Vector Machine, Neural Network, and Decision Tree” are chosen. SPSS has been used to analyze the result regarding the applications of Neural Network helps to diagnose MM.

## 1. Introduction

After the widespread usage of asbestos throughout World War II and subsequently, a significant increase in age-standardized mesothelioma occurrence and fatality rates occurred in the 1960s. The pervasive use of asbestos persisted in high-resource nations (the United States, Europe, and Australia) until the late 1970s and early 1980s when regulatory measures were enacted to limit and prohibit the advertising use of six of the approximately 400 inorganic mineral fibres found in nature “(amphiboles fibres (crocidolite, actinolite, tremolite, anthophyllite, and amosite) and serpentine fibres (chrysotile))”. These six fibres were generally referred to as “asbestos” for legal reasons. The remaining 400 mineral fibres are unregulated, and may be used openly, even though many of them are carcinogenic, and have been linked to mesothelioma. Furthermore, germline mutations in the BRCA1-associated protein 1 (BAP1) and other tumour suppressor genes have been causally related to mesothelioma, sometimes in combination with asbestos or other carcinogenic fibres (gene-environment interaction (GxE)). In addition, therapeutic ionising radiation to the chest, which is typically used to treat lymphomas, has indeed been related to mesothelioma (and sarcomas) in young children [1]. Being exposed to asbestos is the main risk factor for mesothelioma. Up to 80% of all instances can be attributed to it. Asbestos fibres can transfer on skin and clothing, thus living with someone who works with it may raise a person's risk of developing mesothelioma. Some toxins alter a cell's DNA to produce cancer. Others cause cancer indirectly, without directly affecting DNA. For instance, they may speed up cell division, which could enhance the likelihood that DNA modifications will take place. Despite extensive diagnostic workup, the tumour is not a known primary tumour (CUP) metastatic tumour where the primary tumour cannot be identified. CUP represents 1% to 2% of all metastatic tumours and presents a diagnostic and therapeutic challenge. Indirect “platinum-based chemotherapy” is a common first-line treatment, with a response rate of 30% and a “median survival of 9 to 12 months,” respectively. No grading method exists for cancer with an unknown primary (CUP). This is due to cancer already has progressed and the location of the primary cancer's genesis is unknown. CUP can typically be divided into groups by the type of cell that gave rise to it. The aim may be to temporarily reduce the size of the cancer in an effort to alleviate symptoms and lengthen your life because CUP is too developed to be cured. So, the goal of this treatment is to alleviate symptoms like pain rather than to treat the illness, it is referred to as palliative care or supportive care. In recent decades, great efforts have been devoted to identifying the genetic and transcriptional structure of CUP to identify and characterize major molecular changes and gene expression patterns for specific cell-based therapy. Previously, microarray data have been used for DNA and RNA sequencing (RNA-seq), DNA methylation, and whole genome sequencing, with varying degrees of efficiency [2]. Due to issues of distribution, cost, and lack of standardization, such systems are not yet widely integrated into the current CUP analysis workflow.

Therefore, current guidelines for treating CUP still rely on clinical chemistry and immunosuppressive properties to identify the source tissue, 1 although many cases remain undiagnosed and are often treated with therapeutic agents. The use of gene expression data to assess progenitor cells has been extensively studied in the past and RNA-seq methods are more powerful than microarrays in terms of tumour characteristics and diagnostic accuracy. However, due to the large amount of information generated during whole transcript sequencing, it is difficult to develop appropriate analytical methods. Artificial intelligence and machine learning technologies have recently made it possible to analyze large amounts of high-resolution molecular data. Pleural mesothelioma involves “two lung tissues, the viscera of the thorax and the pleura,” accounting for approximately 75% of all mesotheliomas. It develops in the thin membrane that lines the chest cavity and lungs, the pleura. This generally occurs when asbestos fibres get lodged in this lining leading to scarring and inflammation, and subsequently the disease. Pericardial mesothelioma is a type of mesothelioma that involves the mucosa of the pericardium and the mucous membrane that surrounds the heart. It has only been diagnosed in fewer than 200 people in history and this is difficult to research on. The tumours in this cancer form in the lining of the heart, pericardium, and generally results from the metastasis of cancer from another part of the body. Pericardial mesothelioma is often misdiagnosed before autopsy [3]. “Mesothelioma” is always a tumour, but some people may have symptoms of mesothelioma and pleural effusion from mesothelioma. “Severe pain, shortness of breath,” “cough,” “painful and dry cough,” “pleural effusion,” “chest pain,” and “shoulder pain” were common diagnostic symptoms. Other symptoms that may occur in the final stage are weakness, fever, vomiting, high blood pressure (low oxygen in the blood), dysphagia (difficulty in swallowing), fever, night sweats, and weight loss. Clinical characteristics, associated with symptoms, provide measurable information to facilitate assessment. Clinical characteristics such as “histological substructure,” “time to diagnosis,” “platelet count,” “haemoglobin,” and disease levels are used to evaluate survival outcomes according to current methods. In the case of mesothelioma, the industrial history can be very important because it indicates prior asbestos exposure. The risk of developing mesothelioma increases with continued asbestos exposure. Thrombocytopenia can be identified by imaging and diagnostic equipment, including X-ray, MRI, and positron emission tomography (PET). To detect mesothelioma, routine blood tests are necessary [4]. The area that is impacted by MM can be seen on a PET-CT scan. It can also demonstrate whether MM has migrated to the neighbourhood lymph nodes. In rural places, medical imaging technology is pricy and scarce, if it is even accurate and useful. Additionally, a clinical diagnosis like lymphoma is challenging and unsuitable for people. Researchers have used machine learning techniques to solve health information classification problems to speed up diagnosis and simplify testing. “Machine learning” algorithms can collect, process, and analyze medical data in seconds or minutes. X-rays are used in computed tomography (CT) examinations. Magnets and radio waves are used in magnetic resonance imaging (MRI) scans. Both generate static photos of bodily parts and organs. A radioactive tracer is used in PET scans to demonstrate how an organ is operating in real time. The internal organs and tissues of your body are depicted in great detail by a CT scan. A PET scan can be more precise than other imaging procedures and can detect aberrant activity. Additionally, it can cause your body to alter sooner. PET-CT scans are used by doctors to reveal more details about the cancer.

People with “non-mesothelioma” mesothelioma have symptoms similar to mesothelioma, such as pleura. However, these patients were not diagnosed with mesothelioma by their doctors. Clinically it can be difficult to distinguish between “mesothelioma” and “asbestos” patients with pleural effusion and clinical signs suggestive of “mesothelioma” but without the disease. This process can cause breast epithelium, “pleural effusion,” and “other radiological changes” similar to “mesothelioma.” Technical methods for predicting cancer are well known in scientific research. The mesothelioma data used here comes from previous experiments using the probiotic nervous system (PNN) to diagnose mesothelioma. Probabilistic neural networks have also been used to predict responses to chemotherapy and identify future cancer patients. Scientists began their research on simulating probabilistic neural networks, by comparing various “machine learning” algorithms such as “random neural networks,” “random trees,” “decision trees,” and “uniform rules” reproductive power. The design has been written using original databases. These methods were chosen because they are particularly suitable for databases that have been developed by researchers and have previously been shown to be effective and efficient in solving similar health information problems [5]. For example, systems “artificial neural networks” have been used to detect microscopic images of breast cancer and identify specific sequences of “DNA-binding” and “RNA-binding proteins.” Random trees have also found many uses in bioinformatics and psychoanalysis, such as data classification. Researchers have also utilised the random forest to sort data from various malignancies, including lung and renal cell carcinoma. Despite the fact that many mechanical engineering specialists advice beginning with basic mechanical engineering techniques like systematic regress, scientists avoid this since it can be erroneous even when it can be utilised successfully in close settings [6]. The mesothelioma database includes nearly identical datasets derived from similar clinical trials. The researchers used a random tree to extract these features and classify them to identify patient symptoms and clinical predictors of mesothelioma.

Overall, this research presents an argument for the utility of Artificial Intelligence and Machine Learning applications in increasing the accuracy of the early diagnosis of mesothelioma. Such applications will reduce the time taken to analyze the bulk data generated during the mesothelioma diagnosis tests and act in a supportive role to the medical professions. A literature review followed by the use of algorithms to analyze data and a discussion of the generated results comprises the research.

The remainder of this paper is organised as follows.  Section 2 presents a literature review, the methodologies are presented in Section 3, and the results are analyzed in Section 4.  Section 5 contains a discussion of the current work's findings, and Section 6 contains concluding remarks as well as future research directions for the research effort described in this article.

## 2. Literature Review

Malignant mesothelioma (MM) is a malignancy that is rare yet deadly. The number of patients with MM is identified at an elevated level, and the disease is unresponsive to existing treatment methods such as chemotherapy, surgeries, radiation, and immunotherapy. Following a diagnosis of advanced MM, the expected median overall survival is one year. MM has a significant link to asbestos exposure, a material that was widely utilised in the 1970s and 1980s all over the world. Even though asbestos usage was outlawed in the twenty-first, throughout the twentieth century, the “estimated incidence of MM” has consistently climbed due to the disease's long latency period.

Histopathology along with clinical and radiological findings are used to diagnose MM. “Correct diagnosis of MM” is an important step towards successful treatment and has important “medical and legal implications” due to the “problems of profitability” associated with this diagnosis. However, making a clear “MM diagnosis” can be difficult, especially in the early stages. This is often due to symptoms of other malignancies (mainly adenocarcinoma) or the presence of benign/aggressive actions. While the prevalence of MM is decreasing, the goal of early cancer diagnosis is to identify symptomatic individuals as soon as possible to provide them with the greatest chance of obtaining a successful course of treatment. A reduced chance of survival, more treatment-related issues, and higher cost of care are all consequences of delayed or inadequate cancer therapy. A precise diagnosis to avoid complications and speedy deterioration, early detection of diseases to enable speedier intervention and save precious time. All dementia illnesses do not develop in the same way, therefore an accurate diagnosis is helpful in determining the patient's best course of treatment. The use of diagnostic systems (DSS) has increased rapidly over the past two decades. “DSS for MM” allows the “pathologist” to quickly see “medical information.” Most importantly, it can reduce pathological differences [7]. Previous research on “computer-aided MM detection” focused mainly on the development of “automated imaging tools” such as statistical algorithms to identify “pleural projections in breast CT images” and its four numbers. Furthermore, since “pleural thickening” does not always indicate. Until recently, there were not many diagnostic options for MM. For DSS to be more accurate, multidimensional data such as clinical, biological, and radiological aspects of MM should be integrated. Multiple myeloma can be diagnosed using a lot of information. Using a Probabilistic Neural Network (PNN), the researchers achieved a classification rate of 96.30%. On the other hand, comparison agents cannot help in the analysis of MM [8]. Techniques for selecting feature can be used to eliminate features from the “basic feature set” that are pointless or useless allowing the analysis model to focus on more diverse features, thereby improving accuracy and reducing learning time [9]. Classification is important for DSS because the analysis is the main classification problem. In the past various machine learning techniques, such as conveyor belts, “excessive learning machines (ELM),” and deep learning, have been used as classification tools to help analyze “(DL; also called advanced learning). DL makes it easy to create “data views” and different stages of extraction, using algorithms, with many features. Finite Boltzmann machines, automatic coding, “deep belief networks,” and “oscillation neural networks” are all part of this set of DL algorithms [10]. Sound recognition, object recognition, and visual fields are greatly enhanced by these tasks. It has been noted that neural networking-based models that use AI and machine learning are matching or exceeding the accuracy and expectations of results from traditional methods of diagnosis of MM. Thus, it can be said that shifting toward this method is a viable path in the future.

## 3. Methodology

Firstly, the researcher of this paper used MATLAB software to feed the input variables and determined the encoding length. ReliefF and (Genetic Algorithm) GA were used in the MATLAB software to understand how the training and assessment data help the algorithms to become developed. The justification for using the ReliefF method is the efficiency it shows when working with regression problems that have bulk data and improves the result. The implementation of GA will further enhance the quality of solutions to the research problems and optimize the results. Due to the focus on the accuracy of results, these two models were selected for analysis. A total of 70% of the training dataset and 30% of assessment datasets were utilized to develop the diagnostic algorithm for the disease. In this aspect, interpretivist research philosophy was followed to draw the discussion based on the interest of the researcher. Although part research was analyzed, however, the cross-validation folds, number of generations, encoding length, and iterations were selected only by the researcher.

A total of 15 experiments were performed using the two algorithms. GA optimization helped to collect the genetic data of the selected population, and contrarily, it helped to collect the fitness data as well. A ReliefF algorithm was used to select the feature of the disease. The filtering method was used to extract the subsets. The crossover rate of the method was 2 and a significant number of cross-validation folds, iteration numbers, population size, encoding length, number of generations, and number of samples was considered for the experiment.

The accuracy of the current model was obtained 15 times as the experiment was conducted 15 times by changing the number of cross-validation folds, generation number, encoding length, number of runs, and iterations. After that, the set of 15 findings was stored in a Microsoft Excel. Graphical representations were made using the Excel tool and further data analysis was done using “Statistical Package for Social Sciences” or IBM SPSS version 26 software. Descriptive Statistical analysis and multiple regression analysis were carried out with a 95% confidence level. The independent and dependent variables for multiple regression analysis are as follows: *independent variables*: encoding length/number of input variables, cross-validation folds, number of generations, number of iterations, and number of runs. On the other hand, the *dependent variable* is model accuracy. The model accuracy of the technique will help to understand the reliability and the findings of the primary method will be discussed using the recently available journal articles.

## 4. Findings and Analysis through SPSS

The data representation in Table 1 shows the descriptive statistics output where it can be observed that a total of 15 experiments were performed and none of those is missing.

The maximum and minimum numbers of input variables/encoding lengths are 34 and 2, respectively. A maximum of 14 cross-validation folds, 323 iterations, 8 runs, and 100 generations were selected to observe the change in accuracy. It can be observed that the current machine-learning model consisting of the two algorithms is 99.78% accurate (maximum).

Table 2 shows the regression analysis at a 95% confidence level and according to the data, the significance value for “number of encoding variables and coding length” and “model accuracy” has been observed at 0.013 which shows a statistical significance (*p* < 0.05). Again, the value of cross-validation folds and “model accuracy” has been observed at 0.007, which shows a high statistical significance value. The value between the number of generations and model accuracy is 0.013, which shows statistical significance. The significance value between iterations and model accuracy is 0.032, which again shows a high statistical significance. However, the significance value between the number of runs and total model accuracy has been observed at 0.292 which shows a low “statistical significance” or statistically not significant (*p* > 0.05).

This shows that as the number of input variables and encoding length, cross-validation folds, iterations, and the number of generations increases, the overall model accuracy also increases. On the other side, as the number of runs increases, the model accuracy decreases.

Table 3 shows the value of ANOVA regression analysis, and according to the results, the *F* statistics value has been observed at 52.312, which is a high value. Again, the statistical value has been observed at 0.000, which shows a high statistical significance. Thus, the ANOVA regression analysis has shown that the model accuracy has a statistically significant relationship with all the independent variables including the number of runs. This shows that the statistical significance between model accuracy and the number of runs is low statistical significance.

Table 4 shows the model summary of ANOVA regression, and according to the data, the *R* value has been observed at 0.983 and the *R* square value has been observed at 0.967. The adjusted *R* square value has been observed at 0.948. These high values indicate statistical significance. The standard error has been observed at 0.52737.

Figure 1 shows the graphical representation of the relationship between the number of variables and the classification accuracy. According to the data, as the number of input variables increases, the overall classification accuracy also increases.

Figure 2 shows the graphical repression of the relationship between model accuracy and cross-validation folds. According to Figure 2, as the number of cross-validation folds increases, the overall model accuracy also increases.

The regression ANOVA has shown that the cross-validation fold and model accuracy has the highest significance level (0.007). This shows that cross-validation folds have a high degree of relationship with the model accuracy. It can be stated that while implementing “neural networking” for cancer detection, individuals should enhance the number of cross-validation folds. This helps in improving the accuracy level. Thus, medical and healthcare professionals can detect the presence of oncogenic tissues more accurately and rapidly. This on the other hand also would enhance the rapid diagnosis, which will ultimately alleviate the patient's well-being. Therefore, it can be stated that neural networking and cross-validation folds are essential for the proper detection of oncogenic tissue and cell.

## 5. Discussion

Input, secret, and input elements form an autoencoder, a type of three-layer “neural network.” Create a basic encoder using the “encoder” and “decoder” parameters. “Sparse Autoencoder (SAE)” is an autoencoder variant that adds the need for hidden units. The policy includes the following actions:

The following settings are made to the first autoencoder: utilising raw data, concealed image size = 30, hidden image size when using distorted data = 20, standard weight function = 0.001, stop normal function = 4, and spread. Threshold value = 0.05 when the collected data is used as input data for the calculation of the explosion. The parameters of this second autoencoder are hidden representation = 10, control weight for loss = 0.001, delay correction for loss = 4, and scattering ratio = 10. In addition, a linear transmission function is used in this study.

### 5.1. Success Rate

Complexity matrices are used to assess the understanding, specificity, validity, and reliability of each standard procedure and to select the best type of analysis. Since accuracy and precision are often different, the *F*-test is used to measure values and averages F = (accuracy 2)/(accuracy + accuracy).

The performance of the analysis algorithm was evaluated using the receiver's performance characteristic curve (ROC) and the area under the ROC curve (AUC). An efficient way to assess the receiver operating characteristic (ROC) curve, which is described as a graph showing sensitive to a number as the *y* coordinates vs. its favoured or false true positives (FPR) as the *x* coordinates, is used to evaluate the efficacy of diagnostic tests. The ROC test was used to assess the ability of these diagnostic methods. All results were calculated using equations from previous studies [11]. In addition, CPU hours for the SSAE, GA + SSAE analyzers were calculated and compared to show the computing power of each method.

### 5.2. Preprocessing of Data and Feature Extraction

Qualified pathologists divided the entire dataset into two groups: 97 patients with MM and 227 normal individuals. There were 34 variables collected for each individual, and no data was missing. The variety of characteristics may cause a model to be overtrained. As a result, the selection of features is a common pretreatment strategy it omits unrelated, tenuous, or less racial discriminatory elements [12]. The reliability of the generated model can be improved by selecting features. To accomplish feature selection, several feature selection techniques have been created before. GA and ReliefF algorithms were used in this study. These are the GA parameters: the transition frequency is 2, as well as the number of iterations is 100. The population size is 20, the coding length is 34, and the number of generations is 100. The ReliefF parameters are set as below. To detect highly biased data using ReliefF methods, the total number of iterations was 323 and the total number of adjacent samples was 95. Functions used in four data were randomly divided into training (70%) and test data (30%) to develop these diagnostic algorithms.

### 5.3. Models for Diagnostics Construction

Previous research has shown that determining the most efficient mechanism is not always straightforward. As a result, several diagnostic models must be tested to determine which is the most successful. MATLAB software was used to create several diagnostic models in this work, including BP, ELM, and SSAE. Some properties are provided to identify these devices as inputs. In previous works, the mathematical concept of BP was studied. The following are the BP parameters used in this study: hidden layer size = 50, hidden state transfer function = “tansig,” output layer transfer function = “purelin,” training function = “trainlm,” epoch = 1000, and training function good goal = 0.1 value. The learning rate was 0.1. MATLAB default settings were used for other relevant components. In addition, the ELM method was used for the model identification process. ELM is an algorithm for learning neural networks based on hidden neural networks. By formulating input measurements and hidden observations and test measurements in hidden units and through the Moore-Penrose transformation method, particularly when compared to other designs, ELM can attain a high learning rate and a greater generalisation capability. Malignant mesothelioma (MM) is a rare but aggressive form of cancer. Successful therapy depends on the accurate detection of MM, which also has important medicolegal ramifications. The combination epithelial/mesenchymal pattern of MM makes a definite diagnosis difficult. Pleura-related malignancies called malignant mesothelioma (MM) grow in a particularly aggressive manner. Humans exposed to asbestos and asbestiform fibres develop MM. The prevalence of MM is very high.

An earlier study on ELM [13] is available for more information. The number of concealed connections in this investigation is fixed at 30 and the sigmoid value is used as a transfer function. SSAE is a neural network that provides several automatic masks. In this document, two autoencoders are superimposed to produce SSAE to reduce the angle and obtain a high-quality signal without an input signal. When using SSAE, the first autoencoder function is used to obtain the hidden device for the second autoencoder. When the first autoencoder reaches the expected error rate, the next autoencoder generates a higher error rate [14]. In this study, a softmax classification model (SMC) was added to the trained SSAE algorithm to identify classification models. The high-resolution functions obtained by SSAE are used as input to the softmax layer to reset the SMC. SSAE increased in SMC after deep training of the neural network (Figure 3). The previous study of SMC Ken GA and ReliefF reiknir in this study was performed using Software from Numerical computing, Natick, Massachusetts, USA, MATLAB (R2016b 9.1.0.441655). These are the GA parameters: again, the frequency is 2, plus larsä eraður is 100. The population is 20, the coding length is 34, and the gende larði is 100. The ReliefF parameters are set as follows. For the random dataset using the ReliefF method, the number of replicates is 323 and the total number of continuous samples is 95. The models used are randomly divided into four datasets as well as training (70%) and testing (30%) the data for the development of an essay analysis algorithm.

Some tetars are designed to stop the torture. BP's mathematical reasoning was blamed for the interruption. The BP variables used in this study are latent $\text{lagg}\overset{{}^{\circ}}{\text{a}}\text{r}ð\text{t}=50$, latent utslagslagsfústriksfall = “tansig,” uttalskslagfústriksvirkni = “purelin,” training load = “trainlm,” duration = 1000, and target value for the training load = 0. The ratio thereof is 0.1. MATLAB autofocus models are arbitrary for other associated accounts. In addition, the ELM method is used for modelling. ELM is a method of neural learning based on layers of neural networks. Without a system for controlling the input weight and falnum cases and the pregoganum and falnum units in the weight county usually jahverfu Moore-Penrose furlinu, ELM is capable of accelerating acquisition and better performance of the algorithm, especially compared to other data processes. Technical model. You can do preliminary research on ELM [13] to find out more. In this, 30 concealed cells are used in the investigation, and the sigmoid value is used as a control function. SSAE is a neural network system that has many independent inputs. In this paper, two layers of laminate are placed to form SSAE to reduce the angle and obtain high-level properties without input signal.

The parameters of the first autoencoder are determined as follows: hidden image size =30 when using raw data, hidden image size =20 when using data collected by the detrending calculation, standard deweighting operations =0.001, function of normal loss =4 and scatter. Ratio =0.05 when data collected for trend reduction calculations are used as input. These are the parameters of the second autoencoder: hidden representation size =10, weight control for loss =0.001, sparsity correction for loss =4, and sparsity ratio =10 Additionally, linear transfer functions were used in this study.

### 5.4. Success Rate

Confusion matrices were used to evaluate the sensitivity, specificity, accuracy, and reliability of each standard method and to select the most appropriate analysis model. Since sensitivity and precision often separate each other, the *F*-test was used to measure values and averages: *F* = (2 precision sensitivity)/(precision + sensitivity).

The performance of the analysis algorithms was evaluated using the receiver operating characteristic (ROC) curve and the area under the ROC curve (AUC). The effectiveness of these diagnostic methods to distinguish among MM and healthy people was assessed using the ROC test. All results were calculated using standard equations from previous studies [11]. In addition, the CPU hours of the SSAE, GA + SSAE analyzers were calculated and compared to show the computational power of each method. The diagnosis of medical pictures using the visual inspection approach is a time-consuming and subjective operation. Doctors' expertise is useful in the decision-making process. In this way, “image processing algorithms” and machine intelligence technologies avoid diagnoses from being influenced by medical judgments, such as “computed tomography evaluations.” In two phases, the computer-based approach proposed in quickly recognises pleural outlines and identifies pleural glandular tissue. They initially identify the thorax before removing the air and tracheal. They used 3D morphological procedures in both phases. According to the study, using an image processing system to evaluate MM is a potential way to identify the condition. The execution of the randomized walk-based segmentation technique has been found. They attempted to automate the classification of “mesothelioma computed tomography image” collections. To determine the therapies, they used volumetric evaluations to track the disease's course. On PET scans, a 3D variant of the random walk-based segmentation technique may be identified, which is comparable to this technique [15]. They wanted to improve the success rate of lung tumour identification. Rather than using photographs, Er et al. employed numerical information. To be used in the diagnosis of MM disease, “probabilistic neural networks (PNN)” were adapted. Vector quantized neural network-based with several layers were used to compare the findings. With 96.30% accuracy, PNN has been deemed the top classifier. They studied the characteristics of the pleura in both healthy and sick people. They were possible to perceive the thickenings by comparing tracings. By using the 3D “Gibbs-Markov random field (GMRF),” they were able to create a tissue-specific segmentation. It is used to tell the difference between thickenings and thoracic muscle. Then, 3D modelling is used to conduct morphometric evaluations and volumetric evaluations. As per the findings of the study, the automated technique can assist clinicians in diagnosing pleural mesothelioma at a preliminary phase. In another research, gene-expression microarray data were classified using “Principal Component Analysis (PCA)” and the “Brain Emotional Learning (BEL)” network. “Small round blue cell tumours (SRBCTs),” “high-grade gliomas (HGG),” and lung, colorectal, and breast cancers are all classified using the suggested approach combination. The lung cancer dataset includes reports of “malignant pleural mesothelioma.” An uncommon cancer that develops around the chest and lungs is called pleural mesothelioma. Mostly, cases are caused by asbestos exposure. The pleura are malignant (cancerous) pleural mesothelioma develops. This delicate tissue membrane surrounds the lungs and lines the chest walls. A very rare kind of cancer known as pericardial mesothelioma develops in the pericardium, the lining of the heart. Heart (cardiac) tumours are quite uncommon. When they develop, metastasis from cancer in another part of the body is frequently the cause. The PCA–BEL categorised the information with a mean response rate of 100%, 96%, 98.32%, 87.40%, and 88%, as per the findings [16]. For the mesothelioma dataset, numerous “machine learning” methods are already in use. Other strategies, on the other hand, may improve categorization results. As a result, this work tried multiple machine learning approaches on the mesothelioma dataset. Methods were chosen since they had never been used on a dataset previously. As a result, if more precise findings are obtained, the procedure can be employed for advanced diagnostics. In this research, five basic categorization systems are put to test. Techniques are the two types of learning methods. The following subsections provide brief explanations of the methods employed and the parameter setup. In the literature, classification is used to describe a large number of machine learning methods and their variations with different indicators [17]. The majority have been heavily adjusted for biomedical applications. Appropriate outcomes allow for a more in-depth and relevant assessment. In this sense, three basic machine learning approaches have been applied to the mesothelioma database. (a) Support Vector Machine (SVM) is a popular classification method that excels with large datasets and yields more precise results. This can be accomplished by an even small electric locomotive using a “well-fitted optimisation” strategy in kernel mode. Kernel-based modelling is the central element of SVM. To use a kernel function, it divides the data in a high-dimensional feature set. Kernel-based models are preferred due to their efficiency, giving greater results in much less time than other models. This is relevant in MM investigation due to the bulk data produced in the process. Over the ideal hyperplane, SVM produces a decision matrix among samples of various classes [18]. SVM can classify two class datasets into binary categories. The most common methods in fiction are “one versus one” and “one against all.”

Due to the presence of the 2 classifications in the databases, researchers utilised a “one versus one” technique in the research. Various kernels, penalties, and kernel parameters are tried in the beginning phase of the study to determine “well-fitted SVM” configurations for the “mesothelioma datasets”. The findings of all variable tests are listed in Table 5. (a) Decision Tree (DT) is a rule-based machine-learning approach. It is primarily based on tree nomenclature. The rule's determining factor is “information gain (IG).” The categorization is considerably easier to comprehend than previous approaches. It can help with some recurring issues. DT, on the other hand, performs poorly on big databases with few training examples as compared to SVM. Another stumbling block to avoiding overfitting is the trimming procedure. The results of early tests on parameter choices. (d) “Multilayer Perceptron Neural Networks (MLP)”. The enhanced form of NN is the “Multilayer Perceptron (MLP).” Two layers with two components should be used at the very least. Experimental studies are used to examine various parameters and functionality. The weight, as well as the bias of the MLP network, is set at 0.8 and 1, correspondingly, as per the findings. (B) Techniques of Ensemble Learning. The ideas of machine-learning techniques have given rise to ensemble methods. The appropriate combination of many machine learning techniques is fundamental to the ensemble. Multilearners congregate in the decision stage for ensemble techniques, rather than just one learner as in traditional methods, resulting in more effectiveness. Started preparing includes categories from “machine learning” such “DT, KNN, and among others.” This study primarily compares the same learning algorithm (“Decision Tree-DT”) configuration were used in “two prediction models,” but different sample selection techniques were used. The ultimate choice of basic learners is determined by majority voting.

- DTs for bagging. Bagging, also known as bootstrap aggregation, is a technique for enhancing categorization by using well-formed train observations. In the literature, it is sometimes referred to as the resampling procedure. Bagging is a technique that distorts a dataset by resizing it and then utilising the resampled trainsets to train the weak classifier. A voting procedure of parameterization causes the sampling to be distorted. Because the sample weights are all the same, trainsets are chosen at random. As a result, various samples are employed repeatedly in the trainset. It ensures that the distribution of data is more diverse. The ultimate conclusion is determined by the average of each base learner's choice
- DTs and “Adaptive Boosting (Adaboost)”. Boosting is a resampling approach that is comparable to bootstrap. The distinction is that whereas bootstrap disregards sample weighting factors

Then, during the second phase, the probability of incorrectly classified data is enhanced, and successive classifiers are trained. Similarly, other weight factors are used to maintain additional phases [19]. A crucial handbook for boosting theorem is recommended to readers. “Adaptive boosting” outperforms traditional boosting approaches and is more resistant to overfitting problems.

(c) Set of data. The dataset was collected from the University of California, Irvine's dataset repository. It comprises of patients' records received from the “Faculty of Medicine at Dicle University.” The abovementioned machine learning approaches were used to acquire and test 324 MM patient information. There are 34 features with multimodal characteristics in each of the 324 samples in the dataset. In the database, there are no “undisclosed” or “missing value” entries. Doctors provide classifications such as unwell and healthy to patients (2 classes).

Three standard machine learning, as well as two ensemble learning approaches, are used to classify the mesothelioma dataset. Within the conventional machine learning idea, the DT, SVM, and NN approaches are chosen. Bagging and Adaboost using the same week (DT) classifier are, on the other side, an ensemble notion. The evolution metrics are evaluated for reliability and “computational time.” Because there are so many patients with MM illness, time complexity becomes a more essential element in future research with more patient records, due to the integration of 34 factors in addition to a large number of individuals. In regards to computing time, only “10-Fold Cross-Validation” experiments are evaluated. The optimal algorithm takes less time to compute and has a high accuracy rate.

Table 6 shows the overall findings. Table 6 shows that basic DT and SVM as standard machine learning ideas, as well as DT with Bagging as an ensemble approach, outperform other techniques with a similar average accuracy of 100%. In general, different-shaped train sets (2-, 5-, and 10-fold) have little impact. Meanwhile, Adaboost, which uses the same kind of DT as the basic learner but a various sampling selection mechanism called weighted resampling, follows all other algorithms. In this respect, selecting train items randomly is a more successful technique for detecting mesothelioma. Due to the large number of features (34 characteristics) used in classification, selecting a sample using the weight factor is ineffective. Bagging, on the other hand, takes extra computing time due to the uneven sample selection procedure. As a result, when compared to DT and SVM, Bagging is not the recommended approach due to the identical accuracy rates. SVM, a popular kernel-based approach, is evaluated with several kernels and settings. In Table 5, the greatest outcomes of each kernel with varied settings are listed individually.

With 100% in all *K* values, the linear kernel produces the best results. The output of an RBF (radial basis function) depends on the size of the training set. With additional training samples, the overall accuracy increased to 100%, however when the train set was lowered, the success rate declined. Aside from the inconsistency of RBF findings, it contains multiple operations, necessitating more time to categorise large amounts of data. Because of the algorithm's convenience and low time complexity, in reality, “Linear SVM” could be utilised to prevent this time-consuming procedure. These kernels are also linked to the size of the training dataset. In addition to poor accuracies, kernel computational time assessments are not far behind linear kernel analysis. To categorise the mesothelioma datasets, SVM should be used with linear Kernel. The findings suggest that big data may provide better outcomes than previous techniques. MLP, or Multilayer Perceptron in Neural Network language, is used as a final technique. MLP often achieves greater accuracies on nonlinear classification techniques, but it does so over the whole dataset. In this sense, outliers can readily reduce algorithmic effectiveness, necessitating additional processing effort, as seen in Table 6. The dataset contains “34 characteristics over 324 occurrences,” resulting in “34-dimension data.” Because of the intricacy of the dataset, MLP yielded a 97% accuracy rate. SVM, on the other side, focuses on samples that are close to support vectors. As a result of its simplicity and use of prearranged information, SVM outperforms MLP.

## 6. Conclusion

Various machine and ensemble learning strategies for detecting mesothelioma illness are explored in this research. In this sense, a widely used database is used to assess the approaches. Researchers earlier published a paper on the categorization of their information using PNN. With a 3-fold classification algorithm, they had a 96% success rate. Researchers also ran an MLP network with 0.8 weight as well as 1 bias element in this investigation and came to the same conclusion. This implies that the testing procedures are similar and equivalent. Other acquired findings, in this sense, represent constant performance. According to Table 6, the standard machine learning techniques DT and SVM, as well as the ensemble learning technique Bagging, are highly biocompatible with the mesothelioma database. The methods effectively produce a categorization efficiency rate of 100%. In comparison, Bagging are easier algorithms that take less time to compute. In this regard, trapping is not recommended. DT, a rule-based approach, fails to solve the huge data challenge. As a result, due to the large number of people who suffer from mesothelioma condition, it is also ineffective in practice. More data is required to generalise the findings. In that case, DT may provide a false diagnosis. As a result of the aforementioned conclusions and reasoning, linear SVM may be preferable to use in practice. Using such an algorithm supported by linear SVM will allow for the early diagnosis and consequently, an expected lower mortality rate for MM in future. The approaches indicated above will be tried on additional collected data in categorization in future research. After that, a more generic diagnosis system may be developed.

## Figures and Tables

**Figure 1:** Number of variables vs. classification accuracy.

**Figure 2:** Model accuracy vs. cross-validation folds.

**Figure 3:** Architecture of sparse autoencoder.

**Table 1:** Output of descriptive statistics.

Critical analysis						
	N	Min.	Mx.	Average value	Deviation from mean	SD^2
Experiment ID	15	1	15	8.00	4.472	20.000
Number of input variables and encoding length	15	2	34	18.87	10.921	119.267
Cross-validation folds	15	0	14	7.00	4.472	20.000
Number of generations	15	1	100	46.80	32.070	1028.457
Iterations	15	10	323	185.60	114.765	13171.114
Number of runs	15	1	8	4.27	2.251	5.067
Model accuracy	15	92.30	99.78	97.1547	2.31835	5.375
Valid N (listwise)	15					

**Table 2:** Regression coefficient.

Coefficients^a^								
Critical analysis		Overall Val		Coefficient	Number	Key determinant	95%	
		Main Val	Err	Beta			Lower bound	Upper bound
1	(Constant)	94.477	.561		168.433	.000	93.208	95.746
	Number of input variables and encoding length	-.481	.157	-2.265	-3.068	.013	-.835	-.126
	Cross-validation folds	2.479	.709	4.782	3.496	.007	.875	4.084
	Number of generations	-.158	.051	-2.181	-3.095	.013	-.273	-.042
	Iterations	.024	.009	1.192	2.541	.032	.003	.046
	Number of runs	-.632	.565	-.614	-1.119	.292	-1.911	.646

^a^Dependent variable: model accuracy.

**Table 3:** ANOVA.

ANOVA^a^						
Model		Sum of squares	Degrees of freedom	Mean square	*F*	Sig.
1	Regression	72.744	5	14.549	52.312	.000^b^
	Residual	2.503	9	.278		
	Total	75.247	14			

^a^Dependent variable: model accuracy; ^b^Predictors: (constant), number of runs, number of input variables and encoding length, number of generations, iterations, and cross-validation folds.

**Table 4:** Model summary.

Model summary				
Model	*R*	*R* Square	Adjusted *R* Square	Std. error of the estimate
1	.983^a^	.967	.948	.52737

^a^Predictors: (constant), number of runs, number of input variables and encoding length, number of generations, iterations, and cross-validation folds.

**Table 5:** SVM results according to using Kernel.

Kernel	Polynomial	Quadratic	MLP	Linear	RBF
10-fold	97,72	88,98	90,93	100	100
5-fold	97,18	88,75	89,21	100	99,84
2-fold	92,40	84,01	86,11	100	99,07
Time	0,186	0,385	0,089	0,095	0,286

**Table 6:** Overall result of the method.

	DT	SVM (linear)	MLP	Bagging	Adaboost
10-fold	100	100	96,87	100	70,54
5-fold	100	100	95,82	100	65,35
2-fold	100	100	94,44	100	68,82
Time	0,019	0,095	13,89	17,52	0,25

## Data Availability

The data shall be made available on request.
